The article "Comparison and Clinical Value of Ciprofol and Propofol in Intraoperative Adverse Reactions, Operation, Resuscitation, and Satisfaction of Patients under Painless Gastroenteroscopy Anesthesia" was published in 2022. Journal: Contrast Media Mol Imaging.

# Comparison and Clinical Value of Ciprofol and Propofol in Intraoperative Adverse Reactions, Operation, Resuscitation, and Satisfaction of Patients under Painless Gastroenteroscopy Anesthesia

**DOI:** 10.1155/2022/9541060

**Published:** 2022-07-18

**Authors:** Xingqu Chen, Ping Guo, Li Yang, Zhuoling Liu, Deshui Yu

**Affiliations:** ^1^The Second People's Hospital of Yibin, Department of Anesthesiology, Yibin, China; ^2^Department of Critical Care Medicine, The 2nd Affiliated Hospital of Chengdu Medical College, Nuclear Industry 416 Hospital, Chengdu 610051, Sichuan Province, China

## Abstract

**Objective:**

To investigate the comparison and clinical value of ciprofol and propofol for painless gastroenteroscopy anesthesia in terms of intraoperative adverse reactions, operation, resuscitation, and satisfaction of patients.

**Methods:**

A total of 96 patients who underwent painless gastroenteroscopy anesthesia in our hospital from June 2021 to January 2022 were enrolled. The cases were randomly assigned into research group and control group. The control group received propofol anesthesia (*n* = 49), and the research group received ciprofol anesthesia (*n* = 47). The patients, physician satisfaction, vital signs, incidence of adverse reactions, anesthetic first dose, additional time, additional dose, total dose, induction time, insertion time, operation time, awake time, orientation recovery time, leaving room time, and injection pain score were compared.

**Results:**

The overall satisfaction of the study group was higher than that of the control group (*p* < 0.05). After taking medicine, the score of 1 min and MAP in the study group were higher than those in the control group. The incidence of adverse reactions in the study group was lower than that in the control group (*p* < 0.05). The satisfaction of doctors in the study group was higher than that in the control group (*p* < 0.05). The anesthesia induction time, intubation time, operation time, awake time, orientation recovery time, and leaving room time in the study group were significantly longer than those in the control group (*p* < 0.05). The incidence and degree of injection pain in the propofol group were significantly lower than those in the propofol group (*p* < 0.05).

**Conclusion:**

In painless gastroenteroscopy, compared with propofol, ciprofol is equally safe and effective for patients and will not cause early cognitive dysfunction after operation, which is a good choice in painless gastroenteroscopy anesthesia. In addition, ciprofol has significant advantages in patient and physician satisfaction, especially in injection pain. This trial is registered with ChiCTR2100045400.

The article "Comparison and Clinical Value of Ciprofol and Propofol in Intraoperative Adverse Reactions, Operation, Resuscitation, and Satisfaction of Patients under Painless Gastroenteroscopy Anesthesia" was published in 2022. Journal: Contrast Media Mol Imaging.

## 1. Introduction

With the development of anesthetic medicine and the continuous updation of anesthetic drugs, the originally painful endoscopic surgery can be carried out under anesthesia [1]. Painless gastroscopy, painless enteroscopy, painless bronchoscopy, and other endoscopy are widely carried out in outpatient clinic at present, and the development of this technology has greatly promoted the satisfaction and comfort of patients [1]. Painless endoscope can make patients receive diagnosis and treatment comfortably under anesthesia and can obviously reduce the discomfort and pain of patients, but because the diagnosis and treatment time of painless endoscopy is short, the frequency is high, the operation is fast, and the patient is in a state of anesthesia, this leads to anesthetic safety events from time to time, so it is necessary for every anesthesiologist to pay attention to ensuring the safe and effective operation of anesthesia in endoscopic examination [2].

Painless gastroenteroscopy has been widely employed to screen stomach, esophagus, duodenum, and colorectal diseases [3]. Due to discomfort or pain, most tests are performed under sedation or pain, and proper sedation can improve the quality of endoscopy [2, 3]. According to different types of surgery, endoscopic sedation can be assigned into mild, moderate, and deep sedation, and moderate sedation is considered to be the minimum requirement for painless gastroenteroscopy [4, 5]. Nowadays, considering other anesthetics, propofol has many pharmacological advantages, such as quick action, short effect, rapid recovery, and less side effects (such as postoperative nausea and amnesia) [6]. Therefore, the anesthesia of painless gastroenteroscopy mostly uses propofol combined with some sedative and analgesic drugs, and the administration of propofol also chooses intermittent injection. However, due to the individual differences, this mode of administration is easy to cause a transient increase in blood drug concentration in some patients, resulting in respiratory inhibition, and may also cause insufficient depth of anesthesia in some patients, leading to a body movement reaction, which makes endoscopic examination impossible to be carried out smoothly and also reduces the satisfaction of endoscopic physicians and patients [7]. In addition, propofol is easy to cause obvious injection pain at the injection site of the patient, which significantly limits the clinical use of propofol [5]. Our goal is to achieve rapid and predictable recovery, stable cardio-cerebrovascular response, smooth awakening, and less postoperative nausea, vomiting, and other adverse reactions especially with injection pain [8].

The article "Comparison and Clinical Value of Ciprofol and Propofol in Intraoperative Adverse Reactions, Operation, Resuscitation, and Satisfaction of Patients under Painless Gastroenteroscopy Anesthesia" was published in 2022. Journal: Contrast Media Mol Imaging.

Ciprofol is a new intravenous anesthetic developed in recent years, which has a chemical structure similar to that of propofol and thus has similar pharmacological functions to propofol, which has been shown in preclinical experiments with a quick start of action and rapid healing process [9–11]. It is especially noteworthy that at the same used and similar concentrations, the study found that the available dosage form of ciprofol in the aqueous solution was lower than that of propofol, implying that pain injection may be lowered [12, 13], showing a good potential for use, but so far, how effective ciprofol is in painless gastroenteroscopy remains unclear. Based on this, the purpose of this research is to explore the comparison and clinical value of ciprofol and propofol for painless gastroenteroscopy anesthesia in terms of intraoperative adverse reactions, operation, and patient resuscitation and satisfaction, especially the difference in injection pain.

## 2. Patients and Methods

### 2.1. General Information

A total of 96 patients who underwent painless gastroenteroscopy anesthesia in our hospital from June 2021 to January 2022 were enrolled. The cases were randomly assigned into control cohort and research cohort. The control cohort received propofol anesthesia (*n* = 49) and the research group received ciprofol anesthesia (*n* = 47). All patients were asked for medical history in detail before examination, and routine ECG examination, blood pressure measurement, and ECG monitoring were performed. The control group was aged 20 – 65 years, the mean age was (43.20 ± 12.29 years old, the height was 145 – 183 cm, the average height was 160.26 ± 8.47 cm, the weight was 40 – 95 kg, the average weight was (60.74 ± 12.46) kg, the BMI was 17.63-29.75 kg/m2, the average BMI was (23.46 ± 3.43) kg/m2, of which 17 males and 32 females, and 6 ASA Class II cases. There are 43 cases in class I. The age of the study group was 22 – 59 years old, the average age was 41.22 ± 11.63 years old, the height was 150 – 178 cm, the average height was 165.33 ± 7.75 cm, the weight was 43 – 88 kg, the average weight was (60.25 ± 11.22) kg, the BMI was 18.13 – 11.25 kg/m2, the average BMI was 25.22 ± 10.12 kg/m2, of which 22 were males, 25 females, and 4 cases were ASA Level II and 45 cases were ASAI level. There was no statistical significance in the general data. Our hospital's ethics board has given permission for this study, and all patients voluntarily underwent painless gastroenteroscopy, and the patient and his family signed an informed consent form.

#### 2.1.1. Inclusion Criteria

The inclusion criteria were as follows. Voluntarily signed the informed consent form for this research, the vital signs were stable, between 18 and 80 years old, and gastroenteroscopy or treatment was performed for various reasons (but only diagnostic gastroenteroscopy and simple treatment under gastroenteroscopy, endoscopic submucosal dissection, endoscopic retrograde cholangiopancreatography, and other endotracheal intubation procedures were not included). ASA grade I–III. Patients included in the study are not allergic to anesthetics and there are no contraindications to anesthesia.

The article "Comparison and Clinical Value of Ciprofol and Propofol in Intraoperative Adverse Reactions, Operation, Resuscitation, and Satisfaction of Patients under Painless Gastroenteroscopy Anesthesia" was published in 2022. Journal: Contrast Media Mol Imaging.

#### 2.1.2. Exclusion Criteria

The exclusion criteria were as follows. Unable or unwilling to sign consent forms or unable to follow research procedures; patients with incomplete clinical data; unable to visit or cooperate with examinations regularly; contraindications for painless gastroenteroscopy; anesthetic allergy; illiteracy, color blindness, and hearing or visual impairment leading to inability to cooperate with cognitive function assessment; clear central nervous system diseases, such as neurosyphilis, brain tumor, cerebrovascular accident, and so on. Uncontrollable hypertension and diabetes; psychiatric confirmed diagnosis of mental disorders such as depression, somatoform disorders, psychosis, and so on; liver insufficiency (liver enzymes more than 3 times higher than normal) or renal insufficiency (serum creatinine 133 *μ* mol/L); history of malignant tumors (other than digestive tract); history of intravenous anesthesia or general anesthesia (excluding local anesthesia) in the past 3 months. Recent history of sedation and sleep, antianxiety drugs, and antidepressants.

#### 2.1.3. Withdrawal Criteria

The withdrawal criteria were as follows. Follow-up cannot be completed due to various reasons; major complications such as cardiorespiratory arrest, peritonitis caused by perforation, massive hemorrhage, etc.; general anesthesia or pulse anesthesia is performed again for various reasons during follow-up, for example, postoperative pathology suggests that malignant diseases require time-limited surgical intervention; acute events like myocardial infarct, apoplexy, car accident, and lethal occurrence during follow-up. During the follow-up, major life events lead to temperament change and mental abnormality.

Fully inform the patients of the content and purpose of this research, matters to cooperate with, possible risks, and so on; after the patient is confirmed, sign the informed consent form in duplicate, one to the patient, one to the researcher for the record.

### 2.2. Treatment Methods

Patients in both groups were routinely fasting water before operation, gastrointestinal preparations were routinely performed in the morning of examination, no preoperative drugs were given before examination, venous access was established immediately after entering the examination room, various vital signs of patients were monitored, oxygen inhalation 2 L/min with mask was given, and emergency medicine and anesthetic machine were prepared. The patients in the control group were given 1% propofol 1.5∼2.0 mg/kg intravenous injection before gastroscopy or enteroscopy, and the maximum dose of the first load exceeds 0.4 mg/kg in the study group by weight (kg), and the administration time should be 30 seconds. During the inspection operation, additional doses can be added according to the patient's response. It is recommended that each additional dose should not exceed 0.2 mg/kg, the administration time should be 10 seconds, and the interval between each additional dose should be ≥ 2 minutes. Of note, the injection speed should be slow, about 0.5 ml/s, and the dosage of propofol should be adjusted appropriately for those with physical differences. A total of 2% lidocaine 2∼3 ml was added to propofol to relieve the pain and discomfort during intravenous injection. Endoscopic examination was carried out until the patient's conscious experience vanished, as did the eyelash natural reaction, and after OAA/S ≤ 2, endoscopy was performed. Endoscopy is performed after the natural reaction of the eyelashes disappears, and the patient's blood pressure, ECG, and blood oxygen saturation are closely monitored to prevent accidents. Propofol is no longer added when colonoscopy reaches the ileocecum and no treatment is needed. If the patient has physical movement during the examination, propofol 0.2∼0.5 mg/kg should be added. Dopamine 1∼2 mg was injected intravenously when the blood pressure dropped by more than 30%, and atropine 0.5 mg was injected intravenously when the heart rate was less than 60 beats/min, and the SPO2% was always kept above 95%. After the examination, the patient was sent to the recovery room, when he was fully awake, the OAA/S reached level 5, the vital signs were stable and his speech was normal, and then he could leave under the escort of his family. When the patient recovers, it is necessary to lie still and try not to move. Patients are required not to eat or drink within 2 hours after recovery, and some irritating foods should be avoided, which is not conducive to the recovery of patients.

The article "Comparison and Clinical Value of Ciprofol and Propofol in Intraoperative Adverse Reactions, Operation, Resuscitation, and Satisfaction of Patients under Painless Gastroenteroscopy Anesthesia" was published in 2022. Journal: Contrast Media Mol Imaging.

### 2.3. Observation Index

#### 2.3.1. Satisfaction

The satisfaction of postoperative patients and doctors with anesthesia was recorded. The score is 1–5; the higher the score, the higher the patient satisfaction.

#### 2.3.2. Vital Signs

SBP, DBP, MAP, HR, and SPO2 before and 1 min, 2 min, and 3 min after drug administration were recorded.

#### 2.3.3. Incidence of Side Effects

The incidences of side effects such as dizziness, body movement, hypoxemia, hypotension, arrhythmia, atrial premature, cough, hiccup, mandibular support, postoperative delirium, and apnea were recorded.

#### 2.3.4. Operation Condition

The first dose, additional time, additional dose, total dose, induction time, insertion time, operation time, awake time, orientation recovery time, leaving room time, and injection pain score were recorded.

### 2.4. Statistical Analysis

All the data were processed by IBM SPSS21.0, in which the measurement statistics were presented in the form of a mean Std. Deviation ($\bar{x}\pm s$), using one-way analysis of variance, and the counting data were expressed as absolute values, using *χ* 2 test, and the comparison was adjusted by the Bonfferoni test. The statistical results indicated that *p* value less than 0.05 exhibited statistical significance.

## 3. Results

### 3.1. Comparison of Patient Satisfaction

Firstly, we compared patients' satisfaction between both cohorts: the control group had 10 cases of 3 points, 33 cases of 4 points, and 6 cases of 5 points, while the research group had 4 cases of 3 points, 28 cases of 4 points, and 15 cases of 5 points. The results showed that the overall satisfaction of the study group was higher than that of the control group (*p* < 0.05). All the data results are indicated in Figure 1.

### 3.2. Comparison of Vital Signs before and after Administration

Secondly, we compared the vital signs before and after administration, and there was no significant difference before administration (*p* > 0.05). After administration, 1 min, 2 min, and 3 min, the vital signs of the two groups all fluctuated. Moreover, SBP, DBP, MAP, HR, and SPO2 in the research cohort demonstrated none of distinction between both cohorts (*p* > 0.05) except at 60 seconds, and the study cohort's MAP index was greater than that of corresponding cohort (*p* < 0.05). All the data are shown in Tables 1–3.

### 3.3. Comparison of the Incidence of Side Effects

Thirdly, we compared the occurrences of side effects. In the control cohort, only 18 patients had no adverse reactions, the other 31 patients had adverse reactions such as dizziness, body movement, hypoxemia, hypotension, arrhythmia, atrial premature, cough, hiccup, mandibular support, postoperative delirium, and apnea. The total incidence rate was 63.26%. In the research group, 22 patients had no adverse reactions, while the other 25 patients had adverse reactions such as dizziness, body movement, hypoxemia, hypotension, arrhythmia, atrial premature, cough, hiccup, mandibular support, postoperative delirium, apnea, and other adverse reactions, with a total incidence of 53.19%. The occurrence of side effects in the research cohort was less common compared to the control cohort (*p* < 0.05). All the data are indicated in Figure 2.

The article "Comparison and Clinical Value of Ciprofol and Propofol in Intraoperative Adverse Reactions, Operation, Resuscitation, and Satisfaction of Patients under Painless Gastroenteroscopy Anesthesia" was published in 2022. Journal: Contrast Media Mol Imaging.

### 3.4. Comparison of Doctors' Satisfaction

Next, we compared the satisfaction of doctors. In the research group, there were 2 points of satisfaction, 18 cases of 3 points, 16 cases of 4 points, and 11 cases of 5 points. 0 cases in the control group were scored 2 points, 17 cases were 3 points, 27 cases were 4 points, and 5 cases were 5 points; in addition, satisfaction was higher in the study group compared to the control group (*p* < 0.05). All the data are indicated in Figure 3.

### 3.5. Comparison of Induction Time, Insertion Time, Operation Time, Awake Time, Orientation Recovery Time, Leaving Room Time, and Injection Pain Score

Next, we compared the induction time, insertion time, operation time, awake time, orientation recovery time, and leaving room time. The induction time, insertion time, operation time, awake time, orientation recovery time, and leaving room time in the research cohort were obviously greater than those in control cohort (*P* < 0.05). All the data are indicated in Table 4.

### 3.6. Comparison of Pain on Injection

In our study, the injection pain occurrence in the research cohort (1, 2.1%) was significantly less than that of control cohort (11, 71.4%). In the ciprofol groups, only 1 patient had pain on injection, and the score was only 1; in contrast, in the propofol group, 35 patients had injection pain, 13 patients with two scores, 2 patients with three scores, 2 patients with four scores, and 3 patients with five scores. Our results exhibited that the incidence and severity of injection pain in the ciprofol cohort were much less than those in the propofol cohort.

## 4. Discussion

Gastroenteroscopy is the main operation in the department of gastroenterology, which can diagnose gastrointestinal diseases under direct vision and carry out endoscopic treatment [14]. Gastroenteroscopy is assigned into ordinary gastroenteroscopy and painless gastroenteroscopy. The former refers to the gastrointestinal endoscopy without the use of analgesics and sedatives, which can lead to more pain in patients, and even some patients have difficulty to tolerate and resist gastrointestinal endoscopy, while the latter includes the management of pain relief and tranquilizer medications to make patients comfortably accept gastroenteroscopy [15]. Painless gastrointestinal endoscopic sedation is divided into deep sedation and awake sedation, deep sedation puts the patient in an unconscious state, pain disappears, protective reflexes are blunted, and requires the operation of an anesthesiologist; awake sedation is the preservation of the patient's consciousness and response to stimuli such as language, the presence of protective reflexes, stable vital signs, and manipulation by a non-anesthesiologist [16]. It is generally believed that conscious sedation can provide appropriate antianxiety, analgesia, and amnesia for most patients, and it is safer than deep sedation. However, deep sedation can inhibit patients' autonomic reflex and body movement during examination, which is beneficial to the smooth diagnosis and treatment of body movement, such as polypectomy and endoscopic submucosal exfoliation. Therefore, the sedation of gastroenteroscopy tends to be deep sedation, escorted by anesthesiologists, and there are technical specifications for the diagnosis and treatment of sedation/anesthesia by digestive endoscopy for reference [17, 18].

The article "Comparison and Clinical Value of Ciprofol and Propofol in Intraoperative Adverse Reactions, Operation, Resuscitation, and Satisfaction of Patients under Painless Gastroenteroscopy Anesthesia" was published in 2022. Journal: Contrast Media Mol Imaging.

Because propofol has good pharmacokinetic characteristics and can take effect and eliminate quickly, it is an ideal drug to induce and maintain intravenous anesthesia [19, 20]. Propofol injection pain is not rare; although it is not a big problem, it has a bad effect on patients. During anesthesia induction in adults, the incidence of propofol injection pain is 28%∼90%, or even more serious, and the incidence in children is 30%∼90%. Injection pain not only affects the hemodynamics during induction but also affects the physical and mental health of patients, especially children. Injection pain can be assigned into immediate pain and delayed pain [21]. Injection pain is associated with prostaglandins, especially prostaglandin E2. Some of the same people tried to push lidocaine, propofol, and lidocaine mixed injection in advance, giving fentanyl, remifentanil, Kaifen, Ramosetron, and other methods, and the effect is not necessarily good [22].

In our study, the injection pain occurrence in the research cohort (1, 2.1%) was significantly less than that of control cohort (11, 71.4%). In the ciprofol group, only 1 patient had pain on injection, and the score was only 1; in contrast, in the propofol group, 35 patients had pain on injection, 13 cases with two scores of 2, 2 cases with three scores, 2 cases with four scores, and 3 cases with five scores. Our results displayed that the injection pain incidence and severity of the propofol cohort were much greater than those in the ciprofol cohort. On the one hand, the significant decrease in injection pain promotes patients' comfort and compliance; it also reduces other operations that clinicians need to take to reduce or avoid injection pain, simplify procedures, and enhance the operation of anesthesiologists [23]. Our results similarly showed this trend, both in terms of patient satisfaction and physician satisfaction, with a greater scoring of the experiment cohort, a result consistent with the result of injection pain showing that a decrease in injection pain can significantly increase patient experience satisfaction.

The article "Comparison and Clinical Value of Ciprofol and Propofol in Intraoperative Adverse Reactions, Operation, Resuscitation, and Satisfaction of Patients under Painless Gastroenteroscopy Anesthesia" was published in 2022. Journal: Contrast Media Mol Imaging.

Under anesthesia, whether or not the patient's vital signs are smooth is the decisive indicator for evaluating whether anesthesia is successful. Based on this, we compared the vital signs before and after administration, and there was no significant difference before administration (*p* > 0.05). After administration, 1 min, 2 min, and 3 min, the vital signs of the two groups all fluctuated. In addition, no differences were observed between SBP, DBP, MAP, HR, and SPO2 between the two groups of patients (*p* > 0.05). Except that the MAP index of the experimental group was higher than that of the control group (*p* < 0.05). Thirdly, we compared the incidence of side effects. Among the control patients, only 18 patients had no adverse reactions, and the other 31 patients had adverse reactions such as dizziness, body movement, hypoxemia, hypotension, arrhythmia, atrial premature, cough, hiccup, mandibular support, postoperative delirium, and apnea. The total incidence rate was 63.26%. In the research group, 22 patients had no adverse reactions, while the other 25 patients had adverse reactions such as dizziness, body movement, hypoxemia, hypotension, arrhythmia, atrial premature, cough, hiccup, mandibular support, postoperative delirium, apnea, and other adverse reactions, with a total incidence of 53.19%. The incidence of side effects in the ciprofol group was smaller compared to the control cohort (*p* < 0.05). The results of our study overall showed that ciprofol, like propofol, showed no statistical difference in the effects on the vital signs indicators of the patients, and like propofol, ciprofol also had a good safety profile and clinical usability.

In addition, it is worth noting that research cohort's induction time, insertion time, operation time, awake time, orientation recovery time, and leaving room time in the research group were obviously greater than those of the control cohort (*p* < 0.05). Nevertheless, the differences in these indicators do not have a significant impact on surgical procedures, and the injection pain of propofol is within the acceptable range of clinical patients.

Cognitive impairment is a serious adverse effect that occurs after intravenous anesthesia, but none of them showed cognitive impairment in our results [24]. In this study, propofol and cyclopropion anesthesia did not lead to postoperative cognitive impairment for the following reasons: propofol dosage is appropriate, and some studies have shown that the effect of propofol anesthesia on postoperative cognitive function in the elderly is significantly correlated with the dose of anesthesia, and high doses increase the incidence of postoperative cognitive impairment in patients [25]. Considering general anesthesia or combined anesthesia, propofol and ciprofol anesthesia alone eliminated the potential effects of other anesthetic drugs on following surgery cognitive component in the aging population. The results indicated that gastroenteroscopy under propofol and ciprofol anesthesia alone did not cause postoperative cognitive impairment, and animal experiments and clinical studies also indicated that propofol and ciprofol anesthesia were compared with inhalation anesthesia [26]. It has better cognitive effect in the elderly and vulnerable brain. Compared with conventional gastroenteroscopy, painless gastroenteroscopy can reduce patients' pain, relieve patients' tension, reduce stress reaction, is safe and effective for patients, and will not cause early postoperative cognitive dysfunction. In addition, painless gastroenteroscopy has a significant advantage in patient and doctor satisfaction. The deficiency of this study is that the sample size is relatively small with certain limitations and the possibility of statistical deviation. In the future, prospective clinical randomized controlled trial studies with bigger sample capacity are expected to verify the results of this study.

The article "Comparison and Clinical Value of Ciprofol and Propofol in Intraoperative Adverse Reactions, Operation, Resuscitation, and Satisfaction of Patients under Painless Gastroenteroscopy Anesthesia" was published in 2022. Journal: Contrast Media Mol Imaging.

In conclusion, propofol and ciprofol anesthesia is a good choice for surgical anesthesia in the elderly. In painless gastroenteroscopy, compared with propofol, ciprofol is equally safe and effective for patients and will not cause early cognitive dysfunction after operation, which is a good choice in painless gastroenteroscopy anesthesia. In addition, ciprofol has significant advantages in patient and physician satisfaction, especially in injection pain. However, it is worth noting that the dosage of ciprofol should be closely monitored during painless gastroenteroscopy to observe whether there is significant reduction of blood pressure and heart rate, so as to avoid adverse consequences.

## Figures and Tables

**Figure 1:** Comparison of patient satisfaction between two groups.

**Figure 2:** Comparison of the incidence of side effects between two groups.

**Figure 3:** Comparison of doctors' satisfaction between two groups.

**Table 1:** Comparison of vital signs between the two groups $\left[\bar{x}\pm s\right]$.

Group	*N*	SBP				DBP			
		Basic value	1 min	2 min	3 min	Basic value	1 min	2 min	3 min
C group	49	135.17 ± 17.3	119.06 ± 29.06	111.00 ± 13.04	110.77 ± 13.29	87.16 ± 11.18	79.77 ± 13.48	73.79 ± 10.74	71.75 ± 10.9
R group	47	127.3 ± 29.33	123.11 ± 2.15	113.62 ± 20.25	112.42 ± 15.13	87.32 ± 10.22	81.24 ± 11.26	76.35 ± 15.25	75.22 ± 11.40
*T*		1.5969	0.7410	0.7568	0.2239	0.0752	0.5786	0.9632	1.7443
*p*		0.11	0.46	0.45	0.82	0.94	0.56	0.3477	0.08

The article "Comparison and Clinical Value of Ciprofol and Propofol in Intraoperative Adverse Reactions, Operation, Resuscitation, and Satisfaction of Patients under Painless Gastroenteroscopy Anesthesia" was published in 2022. Journal: Contrast Media Mol Imaging.

**Table 2:** Comparison of vital signs between the two groups $\left[\bar{x}\pm s\right]$.

Group	*N*	MAP				HR			
		Basic value	1 min	2 min	3 min	Basic value	1 min	2 min	3 min
*C* group	49	100.53 ± 11.92	92.11 ± 12.71	86.22 ± 13.64	82.28 ± 12.14	82.69 ± 15.56	79.46 ± 10.68	77.22 ± 9.20	74.95 ± 9.03
*R* group	47	99.22 ± 10.25	98.22 ± 10.31	87.45 ± 14.28	86.33 ± 13.25	81.33 ± 11.25	78.69 ± 18.32	79.25 ± 14.85	75.96 ± 14.68
*t*		0.5763	2.5804	0.4316	1.5625	0.7528	1.1528	0.7256	0.6582
*p*		0.57	0.011	0.6670	0.1215	0.626	0.8009	0.4207	0.6843

**Table 3:** Comparison of vital signs between the two groups $\left[\bar{x}\pm s\right]$.

Group	*N*	SPO2			
		Basic value	1 min	2 min	3 min
C group	49	99.53 ± 0.84	99.16 ± 1.72	97.85 ± 2.44	98.40 ± 2.37
R group	47	97.63 ± 3.34	99.18 ± 3.39	97.33 ± 4.52	98.22 ± 3.65
*T*		0.4589	0.3655	0.6835	0.7589
*p*		0.23	0.9708	0.48	0.7742

**Table 4:** The different induction time, insertion time, operation time, awake time, orientation recovery time, leaving room time, and injection pain score between the two groups $\left[\bar{x}\pm s\right]$.

Group	*N*	Induction time (min)	Insertion time (min)	Operation time (min)	Waking time (min)	Directional force recovery time (min)	Departure time (min)
C group	49	1.08 ± 0.40	1.40 ± 0.70	4.71 ± 2.09	3.08 ± 2.15	3.69 ± 2.16	6.65 ± 2.78
R group	47	2.98 ± 0.77	3.45 ± 1.03	6.11 ± 2.52	6.22 ± 1.56	6.19 ± 2.36	9.96 ± 3.14
*T*		5.562	6.255	6.785	7.259	5.854	6.351
*p*		＜0.01	＜0.01	＜0.01	＜0.01	＜0.01	＜0.01

## Data Availability

No data were used to support this study.
